# PKCε Activation Restores Loss of PKCε, Manganese Superoxide Dismutase, Vascular Endothelial Growth Factor, and Microvessels in Aged and Alzheimer’s Disease Hippocampus

This article has been retracted.

**DOI:** 10.3389/fnagi.2022.836634

**Published:** 2022-03-01

**Authors:** Guetchyn Millien, Huaixing Wang, Zongxiu Zhang, Dan L. Alkon, Jarin Hongpaisan

**Affiliations:** ^1^Center for Translational Medicine, Department of Medicine, Sidney Kimmel Medical College, Thomas Jefferson University, Philadelphia, PA, United States; ^2^Neurotrope Bioscience, Inc., New York, NY, United States

**Keywords:** aging, Alzheimer’s disease, hippocampus, PKCε, oxidative stress, microvessel

## Abstract

Vascular endothelial dysfunction and capillary loss are currently considered to be a primary phenotype of normal human aging and Alzheimer’s disease (AD). Activation of protein kinase C (PKCε) improves several molecular, cellular, physiological, and behavioral endpoints, yet it is not known whether a loss of PKCε activity occurs in the microvascular endothelium in aged and AD hippocampi, whether this loss contributes to microvascular change, or whether activation of PKCε protects against microvascular damage, an early change that induces age-associated memory defect and AD. We investigated the effect of the PKCε activation on microvascular loss in the hippocampus, important for memory storage. In cultured human brain microvascular endothelial cells, tert-butyl hydroperoxide induced oxidative stress and a decrease in manganese superoxide dismutase (MnSOD) mRNA and protein expression that were blocked by the antioxidant drugs. The PKCε activators bryostatin and DCPLA methyl ester increased PKCε, associated with an increase in MnSOD mRNA and its protein as well as vascular endothelial growth factor (VEGF), which was inhibited by the mRNA-stabilizing HuR inhibitors. In rats (>24 months old) and AD transgenic mice Tg2576 (5 months old), bryostatin or DCP-LA prevented a decrease in vascular PKCε, MnSOD, and VEGF and prevented microvascular loss and age-related memory impairment. An autopsy-confirmed AD hippocampus showed a decrease in PKCε and MnSOD mRNAs and their proteins and VEGF as well as in microvascular density compared to non-AD controls. In conclusion, the PKCε activation can rescue a decrease in PKCε, MnSOD, and VEGF *via* posttranscription regulation and alleviate oxidative stress, and in doing so, prevent microvascular loss during aging and AD.

## Introduction

Cerebral rarefaction of capillaries and terminal arterioles results in reduced microcirculation and hypoxia, often attributed to neurodegeneration and currently considered to be a primary phenotype of normal human aging and Alzheimer’s disease (AD) (Kemper et al., 1999; Riddle et al., 2003; Desai et al., 2009; Arvanitakis et al., 2011; Brown and Thore, 2011; Toda, 2012; Ungvari et al., 2018). In addition, disruption of the blood-brain barrier (BBB) has been shown to prevent the clearance of amyloid beta (Aβ), which is known to increase during aging and AD, not only leading to amyloid plaque deposition, but also an increase in oxidative stress, inflammation, and cerebrovascular damage (Hawkes et al., 2011; Qosa et al., 2014). Moreover, oxidative damage is considered another main driving force in the aging process as well as in AD pathogenesis (Harman, 1956; Nunomura et al., 2001; Sanz and Stefanatos, 2008). Therefore, drugs targeting microvascular (MV) damage and oxidative stress may be candidates for treating age-related memory impairment and AD (Kaan et al., 2013).

The three prime untranslated region (3′-UTR) is the section of messenger RNA (mRNA) that immediately follows the translation termination codon. The 3′-UTR often contains regulatory regions that post-transcriptionally influence gene expression. Protein kinase C (PKC) can activate the nuclear export and transport of the mRNA-stabilizing embryonic lethal, abnormal vision (ELAV), Drosophila -like, or human antigen (Hu) family proteins (HuR, HuB, HuC, and HuD) that will bind with AU-rich (ARE) sequence in the 3′-UTR, resulting in the inhibition of mRNA degradation (Chung et al., 1997; Antic and Keene, 1998; Quattrone et al., 2001; Pascale et al., 2004, 2005). The 3′-UTRs of human manganese superoxide dismutase (MnSOD) and vascular endothelial growth factor A (VEGF-A or VEGF) have multiple ARE sequences (King, 2000; Wang et al., 2001; Chaudhuri et al., 2012; Arcondeguy et al., 2013). HuR protein prevents VEGF mRNA degradation that enhances VEGF protein synthesis in vascular endothelial cells (Arcondeguy et al., 2013).

PKCε and PKCα isozymes may promote the transcription of the mitochondrial antioxidant MnSOD in human lung cells and acute myeloid leukemia (Chung et al., 2011; Di Marcantonio et al., 2018). PKCε can increase expression of VEGF outside of the brain (Amadio et al., 2012). Others have reported that PKCε stimulates cardiovascular endothelial cell proliferation and angiogenesis (Davis et al., 2007); protects against oxidative damage, inflammation, and apoptosis (Chattopadhyay et al., 2014); and supports endothelial integrity *via* tight junctions (Sonobe et al., 2009).

A decrease in PKC activity has also been observed in the aging brain at the level of the whole hippocampus (Battaini and Pascale, 2005; Govoni et al., 2010). Down-regulation of PKCε isozyme occurs at the neuronal cell or structural level in the hippocampal CA1 area in aged rats (Hongpaisan et al., 2013). Synaptic formation in the hippocampal CA1 area is important for spatial memory retention, and synaptic loss in this hippocampus is associated with age-related memory impairment (Hongpaisan and Alkon, 2007; Hongpaisan et al., 2013). Additionally, down-regulation of MnSOD, parallel to elevation of oxidative stress, is evident during aging (El Assar et al., 2013). Loss of PKCε occurs in AD neurons (Hongpaisan et al., 2013; Sen et al., 2018). Activation of PKCε improves several molecular, cellular, physiological, and behavioral endpoints, including degradation of Aβ, prevention of synaptic loss, induction of synaptogenesis, and prevention of cognitive deficits and memory loss (Hongpaisan et al., 2011; Sen et al., 2012).

It is not known whether a loss of PKCε activity also occurs in the MV endothelium in aged and AD hippocampi, whether this loss contributes to MV change, or whether activation of PKCε protects against MV damage, which is one of several early changes that induce age-associated memory defect and AD. In the present study, we studied the effects of the PKCε activator and peroxide tert-butyl hydroperoxide (TBHP)-induced oxidative stress on PKCε, MnSOD, and VEGF in human brain MV endothelial cells (HBMEC) in cultures. We also measured changes in PKCε, MnSOD, and VEGF in microvessels associated with MV density in the hippocampus and the therapeutic effects of the PKCε activators 8-(2-(2-pentyl-cyclopropylmethyl)-cyclopropyl)-octanoic acid (DCP-LA) and bryostatin in age-related memory impaired rats, AD transgenic mice Tg2576, and/or autopsy-confirmed AD human subjects. Change in microvessels was focused in the stratum radiatum of the dorsal hippocampal CA1 area, comprising apical dendrites of the CA1 pyramidal neurons. Changes in dendritic spine morphology and synaptic density in the dorsal hippocampus – particularly the generation of mushroom spines and synapses within the apical dendrites of CA1 pyramidal neurons– are correlated with changes in spatial memory (Hongpaisan and Alkon, 2007).

## Materials and Methods

### Cell Culturing

Human brain MV endothelial cells (Neuromics, Edina, MN, United States, cat # HEC02 or ScienCell Research Laboratories, Carlsbad, CA, United States, cat # 1000) at subculture passage 2–5 were grown on fibronectin-coated cover glasses (0.8 mm diameter) in 12-well plates or fibronectin-coated 6-well plates. Cultured cells were maintained in endothelial medium (ScienCell) supplemented with the endothelial cell growth supplement (ECGS, ScienCell) and 5% fecal calf serum up to 3 days at about 1 ml per well (3.5 cm^2^ surface area) on the 12-well plate or 3 ml per well (9.6 cm^2^ surface area) on the 6-well plate. Because unlike most other cell types, HBMEC could not survive under serum-free medium to induce maturity, the limited culture medium and fecal calf serum, without fresh culture medium change, allowed HBMEC cells to initially multiply and thereafter reach maturity during the gradual exhaustion of serum. For immunohistochemistry, cultured cells growing on cover glasses were fixed with 4% paraformaldehyde at room temperature for 15–20 min and kept in phosphate buffered saline (PBS) at 4°C.

### Measurement of Superoxide

The specific probe hydroethidine (Thermo Fisher Scientific, Waltham, MA, United States, cat # D11347) was used to measure changes in cellular superoxide (O_2_^•–^) production (Sen and Hongpaisan, 2018). The reaction between O_2_^•–^ and non-fluorescent hydroethidine generates a highly specific red fluorescent product, 2-hydroxyethidium. In biological systems, another red fluorescent product ethidium is also formed, usually at a much higher concentration than 2-hydroxyethidium (Zielonka and Kalyanaraman, 2010). Cultured cells, grown on glass slides, were incubated with hydroethidine (2 μg/ml) at room temperature for 15–20 min and then fixed with 4% paraformaldehyde. Increased O_2_^•–^ production was qualitatively determined with a confocal microscope at 488 nm/>510 nm (excitation/emission).

### Aged Rats With Learning Impairment

Brown Norway rats were obtained from the National Institute on Aging, National Institutes of Health (NIH) facilities (Harlan, Indianapolis, IN, United States). Animals were housed in an animal facility for 1 month prior to experiment to recover from transport. Young rats (5 months) and aged rats (>24 months) were trained in a water maze pool, as previously described (Hongpaisan et al., 2013). In short, rats were trained to find a platform hidden by dissolving non-toxic white tempera (BesTemp; Certified Color Corp., Orange, CA, United States) in the water (two swims per day for 5 days). Aged rats were divided into two groups: (1) aged, learning-unimpaired group; and (2) aged, learning-impaired group (Hongpaisan et al., 2013). Only aged, learning-impaired rats were used in the present study. Rats were injected with the PKCε activators (5 μg/kg bryostatin [MilliporeSigma, Burlington, MA, United States, cat # 203811] or 1.5 mg/kg DCP-LA [MedChemExpress, Monmouth Junction, NJ, United States, cat # HY-108599A] diluted with normal saline, i.p., every other day for five injections before and three more injections during spatial memory training), compared to young and aged rats injected with normal saline (in the absence of the PKCε activator). Ten days after the first 5-day swim, rats were trained for the second 5-day swim. At 24 h later, the probe test was carried out to test the memory of rats to concentrate their swimming on the removed platform area.

### Alzheimer’s Disease Transgenic Mice

Male Tg2576 [Genotype: Hemizygous for 129S6.Cg-Tg(APPSWE)2576Kha N20] and wild-type control mice (approximately 2 months old) were purchased from Taconic (Hudson, NY, United States) and housed for 1 week before the experiment to recover from transport stress. Bryostatin, kindly provided by the National Cancer Institute (NCI), NIH (Bethesda, MD, United States), was administered in 2 doses/week for 14 weeks (30 μg/kg body weight, dissolved in sterile normal saline, i.p.). Non-treated groups received the same volume of normal saline, mechanism of delivery, and frequency of administration as the treated groups.

### Animal Brain Tissue Preparation

Rats and mice were deeply anesthetized with sodium pentobarbital (120 mg/kg body weight, i.p.). Animals were perfused through the heart with cold PBS for less than 4 min to wash out the blood and subsequently with 4% paraformaldehyde in PBS. Brains were then removed, postfixed for 20 min, and stored in PBS at 4°C. Under the stereoscope, the right brain was dissected, and the midbrain and cortex part were removed to expose the hippocampus. The right dorsal hippocampus and cerebral cortex were excised. A small piece of filter paper partially wet with PBS was used to remove excessive PBS and to transfer tissue to mount on the vibratome stage with super glue that was spread to a thin layer with another dried filter paper. Using the remaining cerebral cortex as the support, the hippocampus was sectioned with a vibratome (Leica VT1200S; Leica Microsystems, Wetzlar, Germany) into 200 μm (for mouse) or 300 μm (for rat) thickness and kept in series in PBC at 4°C. The hippocampal cross-sections were excised from the serial sections; #1, #4, #7, and #9 (400 μm apart for mouse or 600 μm apart for rat) were further fixed in 4% formaldehyde in PBS at 4°C overnight to harden the tissue. The 200 or 300-μm thickness tissue section was mounted on a vibratome stage with a thin layer of super glue and then cut again with the vibratome into 5 μm thickness by adjusting the suitable knife angle, sectioning arm speed, and vibrating frequency. Four hippocampal sections at 5-μm thickness were then processed free-floating for immunohistochemistry and cytochemistry. A watercolor painting brush #0 trimmed to have just a couple of hairs was used to carry thin tissue sections from the buffer bath of vibratome. Tissue sections (clear of excessive glue) were immersed with the painting brush to attach the container floor without rocking or shaking during antibody incubation or washing to prevent the sections floating on the surface of solution.

### Human Brain Tissue Preparation

The pathological diagnosis of AD was conducted according to the Consortium to Establish a Registry for Alzheimer’s Disease (CERAD). All patients (or relatives/representatives who had the power of attorney) signed informed consent forms. The present work was carried out in accordance with the Code of Ethics of the World Medical Association (Declaration of Helsinki) for experiments involving humans^1^. Autopsied brains were fixed in 10% formalin. Human hippocampal samples at 0.4 cm thickness were processed for paraffin embedding. Paraffin-embedded sections (10 μm) were mounted on glass slides and deparaffinized with xylene (two times; 5 min each) and 100% ethanol for 5 min. Tissue sections were then rehydrated with graded alcohol. For antigen retrieval of human autopsies, deparaffinized hippocampal sections were incubated in 10 mM citrate buffer pH 6.0 added with 0.05% Tween at 95°C for 30 min.

### Immunohistochemistry, Cytochemistry, and Confocal Microscopy

Tissue specimens were treated with Image-iTTM FX signal enhancer (Thermo Fisher Scientific, Waltham, MA, United States) for 30 min and PBS containing 15% serum and 0.5% Triton X-100 for 60 min at room temperature, to block non-specific protein binding sites. For primary antibody incubation, specimens were incubated overnight at room temperature, except that human tissue were incubated at 4°C for 3 days and at room temperature for 24 h. Primary antibodies are anti-PKCε (rabbit polyclonal IgG; 1:100; MilliporeSigma, Burlington, MA, United States, Cat # 06-991), platelet/endothelial cell adhesion molecules-1 (PECAM or CD31, goat polyclonal antibody, Santa Cruz Biotechnology, Dallas, Tx, United States, cat # sc-37664), anti-PKCα (mouse monoclonal IgG; 1:100; MilliporeSigma, Burlington, MA, United States/Upstate, cat # 23336), anti-MnSOD (rabbit polyclonal IgG; 1:100; MilliporeSigma, Burlington, MA, United States, cat # 06-984), and anti-VEGF (mouse monoclonal IgG; 1:50; Santa Cruz Biotechnology, Dallas, Tx, United States, cat # sc-7269). Specimens were then incubated with biotinylated horse anti-mouse antibody (1:20; Vector Laboratories, Burlingame, CA, United States, cat # BA-2000) and/or Alexa Fluor 568 donkey anti-rabbit (cat # A10042) or goat (cat # A11057) antibody (1:200; Thermo Fisher Scientific, Waltham, MA, United States) for 3 h at room temperature. For blood vessel staining, rodent tissue sections were incubated with biotin-conjugated isolectin B4 (IB4) from *Bandeiraea simplicifolia* (*Griffonia simplicifolia*, 1:50; Vector Laboratories, Burlingame, CA, United States, cat # B-1205) at room temperature for 4 h. Tissue sections treated with biotinylated antibody or lectin were incubated with Alexa Fluor 488 streptavidin (1:100; Thermo Fisher Scientific, Waltham, MA, United States, cat # S11223A) for 3 h at room temperature. After each lectin and/or antibody incubation, the samples were washed with PBS three times (each time for a period of 5 min). Sections were mounted with VECTASHIELD mounting medium with DAPI (Vector Laboratories, Burlingame, CA, United States) to counterstain nuclei. For negative controls, primary or secondary antibodies was were replaced with protein with no antigenicity against the tested antibody.

Hippocampal slices were oriented with a Zeiss Axio Observer Z1 microscope equipped with a 710 confocal scanning system using the 10x objective lens in the DAPI channel (for staining nuclei). The random CA1 area that appeared immediately after switching to the higher magnification lens, either 63X or 100x Plan-APO Chromat oil immersion objectives (1.4 NA), was imaged for appropriate fluorescence (e.g., Alexa 488 and/or 568). Confocal images of hippocampal sections were acquired in line scan mode with a pinhole of approximately 1.00 Airy unit and averaged data from several images were reported.

### Quantitative Analysis of Immunohistochemistry

Protein expression was determined with semi-quantitative analysis. All tissue samples within the same experiment were processed for immunohistochemistry at the same time and imaged with the same set-up of confocal microscope (the same objective lens, digital magnification, etc.) within the same day. At least five images were randomly collected from each culture, animal, and human brain. The confocal images were transferred to quantify them in another computer with the ImageJ program^2^. The individual image was collected at 1024 pixels × 1024 pixels. For individual analysis, a group of eight bits was assigned one of the 225 possible integers from 0 to 255 to each pixel. Individual cells were identified with specific immune-expression (Alexa 488 or 568) to stain the target proteins and their DAPI-stained nucleus. The border of each individual cultured cell was rather clear, while the border between two adjacent cells in the *in situ* microvessels was imagined at the middle line between 2 different nuclei. Under ImageJ program, regions of interest (ROI) of each individual cell were manually drawn and analyzed for the mean gray intensity value from the pixels of:

1. Alexa 488 or 568 within the cell area (the cytosol and nucleus together) for target protein, except for mitochondrial MnSOD (only in the cytoplasm), and
2. DAPI within the nuclear area.

Data were collected at a single cell level (Alexa 488 or 568 intensity of the target protein normalized with its nuclear DAPI intensity). Data were averaged from the overall cells collected under the same experiment group. The averaged control data were set at 100%, and all other experiment data were defined as % of their controls.

### Cell Lysis and Western Blot Analysis

Cultured cells were harvested in homogenizing buffer (HB) containing 10 mM Tris-Cl (pH 7.4), 1 mM PMSF (phenylmethylsulfonylfluoride), 1 mM EGTA, 1 mM EDTA, 50 mM NaF, 20 μM leupeptin, and 1% Triton X-100 and were lysed by sonication. Protein concentration was measured using the Coomassie Plus (Bradford) Protein Assay kit (Pierce, Rockford, IL, United States). About 20 μg of protein from each sample was subjected to SDS-PAGE analysis in a 4–20% gradient Tris-glycine polyacrylamide gel (Invitrogen, Waltham, MA, United States). The separated protein was then transferred to a nitrocellulose membrane, blocked with BSA, and incubated at 4°C overnight with primary antibodies: anti-PKCε (rabbit polyclonal IgG; 1:500; Novus Biologicals, Littleton, CO, United States, NBP2-19848), anti-MnSOD (mouse monoclonal IgG; 1:1,000; MilliporeSigma, Burlington, MA, United States, cat # 06-984), anti-VEGF (rabbit polyclonal IgG; 1:500; Invitrogen, Waltham, MA, United States, cat # PA1-16948), anti- β -Actin (mouse monoclonal IgG; 1:25,000, Millipore, MABT825 or rabbit polyclonal IgG; 1:25,000, Novus Biologicals, Littleton, CO, United States, NBP2-7636). After being washed three times with TBS-T (Tris-buffered saline-Tween 20), the membrane was further incubated with alkaline phosphatase conjugated secondary antibody (1:10,000) for 45 min. The membrane was again washed three times with TBS-T and developed with the 1-step NBT-BCIP substrate (Pierce, Rockford, IL, United States). The blot was imaged in an ImageQuant RT-ECL (GE Life Sciences, Piscataway, NJ, United States), and densitometric quantification was performed using Image J software. For quantifying expression of a protein, the densitometric value for the protein of interest was normalized against β-Actin (loading control).

### RNA Isolation and Quantitative PCR

Human brain MV endothelial cells cultured cells from 6-well or p100 plates were washed with 1X PBS followed by trypsinization using diluted trypsin added to each well at room temperature. Cells were observed under a microscope for complete dissociation and transferred to 1.5-ml Eppendorf tubes containing fetal bovine serum and mixed to inactivate trypsin spin at 1000 rpm for 5 min. The supernatants were removed, pellets were washed with 1 ml 1X PBS, 350 μl RLT buffer was added, and the cells were stored at –80 for subsequent RNA isolation. Total RNA was isolated using RNeasy kit with on column DNase treatment following the manufacturer’s protocol. The 1 μg of total RNA was reverse transcribed (RT) using Omniscript (Qiagen, Germantown, MD, United States), and quantitative real-time PCR (qPCR) was performed with FAST SYBR Green or Fast TaqMan master mix (Life Technologies, Carlsbad, CA, United States) on the Step One plus ABI 7000 machine (Applied Biosystems, Waltham, MA, United States). Data were normalized to 18S. PCR assays are:

**Table:** 

**Assay name**	**Assay ID**	**Vendor**
PKC epsilon (PRKCE)	HP208540	Origene
MnSOD	Hs00167309_m1	Thermofisher
B-Actin	Hs99999903_m1	Thermofisher
18S	Hs99999901_s1	Thermofisher
VEGFA	Hs00900055_m1	Thermofisher

### Statistical Analysis

Data with two experimental groups, western blot, and qPCR were analyzed with Student’s *t*-test. For experiments with three or more groups, data with a significant overall difference among the groups as demonstrated by ANOVA were further analyzed by Tukey multiple comparisons. The confidence level was set at 95% (α = 0.05).

## Results

### Effects of the PKCε Activator on the Tert-Butyl Hydroperoxide-Induced Increase in Superoxide (O_2_^•–^) Production

Oxidative damage is the main driving force in the aging process (Harman, 1956; Sanz and Stefanatos, 2008). Stable organic peroxide TBHP was used to induce mitochondrial dysfunction, leading to an increase in O_2_^•–^ and oxidative stress (Elmlinger et al., 2011; Fedotcheva and Mokhova, 2013). Cultured HBMEC cells at 95% confluence were treated with 50, 200, or 500 μM TBHP for 1 h and switched to the fresh culture medium without TBHP for 3 days, compared to control cells treated accordingly without TBHP. Fluorescence imaging of ethidium was used to determine O_2_^•–^ level (Figure 1A). Intracellular O_2_^•–^ level was increased on day 3, but not day 1, in a TBHP concentration-dependent fashion (Figure 1B). TBHP only at 500 μM was then used in later experiment.

**FIGURE 1:** The PKCε activator prevents an increase in reactive oxygen species (ROS) and a decrease in MnSOD mRNA expression and increases PKCε mRNA expression in human brain microvascular endothelial cells (HBMEC) treated with tert-butyl hydroperoxide (TBHP). **(A)** TBHP was used to induce mitochondrial dysfunction and an increase in reactive oxygen species (ROS), including superoxide (O_2_^•–^). Cultured cells were treated with 0, 50, 200, or 500 μM TBHP for 1 h and recovered in new culture medium without TBHP for 1 or 3 days. The reaction between O_2_^•–^ and non-fluorescent hydroethidine generates highly specific red fluorescent products, ethidium and 2-hydroxyethidium (Zielonka and Kalyanaraman, 2010) were used to determine **(B)** concentration-dependent effect of TBHP on intracellular O_2_^•–^ production. **(C–F)** Cells had been incubated with 500 μM TBHP for 1 h and were incubated in fresh culture medium without TBHP in an absence or presence of the PKCε activator bryostatin (bry, 25 nM) or DCPLA-ME (DCP, 100 nM) for 3 days. **(C)** Effects of bryostatin and DCPLA-ME on O_2_^•–^ production, determined by ethidium and 2-hydroxyethidium as in the panel **(A)**. Quantitative PCR (qPCR) was used to determine **(D)** PKCε, **(E)** MnSOD, and **(F)** VEGF mRNA expression. Data are represented as mean ± SEM, *p < 0.05; **p < 0.01; ***p < 0.001; one-way ANOVA and *post hoc* Tukey’s multiple comparison test (*n* = 110–465 random cells from 3 to 4 cultures/group) or Student’s *t*-test for double measurement qPCR (*n* = 4–5 cultures/group).

After 500 μM TBHP for 1 h, cultured HBMEC cells were treated with the PKCε activator bryostatin (25 nM, MilliporeSigma, Burlington, MA, United States) or DCPLA-ME (100 nM, MedChemExpress, Monmouth Junction, NJ, United States) for 3 days, compared with control cells treated accordingly without TBHP and the PKCε activator. As summarized in Figure 1C, bryostatin and DCPLA-ME decreased intracellular O_2_^•–^ level compared to the basal O_2_^•–^ level in cells without TBHP treatment but prevented an increase in O_2_^•–^ level in cells treated with TBHP. The results indicate that PKCε activation can reduce oxidative stress.

### Effect of the PKCε Activator on the Tert-Butyl Hydroperoxide-Induced Change in PKCε, Manganese Superoxide Dismutase, and Vascular Endothelial Growth Factor

Change in mRNA expression was studied with quantitative PCR (qPCR, Figures 1D–F), while protein expression was studied with immunohistochemistry (Figures 2A,E,I) and western blotting (Figures 2C,G,K). TBHP decreased MnSOD mRNA (Figure 1E) and protein (Figures 2E–H) but had no effect on PKCε (Figures 1D, 2A–D) and VEGF (Figures 1F, 2I–L) mRNA and protein expression. The results indicate that TBHP-dependent oxidative stress is correlated with a decrease in MnSOD, but not PKCε and VEGF, mRNA expression and translation.

**FIGURE 2:** PKCε activation increases PKCε, MnSOD, and VEGF protein expression in cultured human brain microvascular endothelial cells (HBMEC) treated with tert-butyl hydroperoxide (TBHP). Cultured cells were treated with 500 μM TBHP for 1 h and incubated in new culture medium with or without the PKCε activators bryostatin (bry, 25 nM) and DCPLA-ME (DCP, 100 nM) for 3 days. **(A,B,E,F,I,J)** Immunohistochemistry imaged with confocal microscopy and **(C,D,G,H,K,L)** western blot analysis of **(A–D)** PKCε, **(E–H)** MnSOD, and **(I–L)** VEGF. M, molecular weight marker. Data are represented as mean ± SEM, *p < 0.05; **p < 0.01; ***p < 0.001; one-way ANOVA and *post hoc* Tukey’s multiple comparison test (*n* = 59–134 MnSOD-immunostained cells or 451–907 PKCε or VEGF-immunostained cells from 3 to 4 cultures/group or t-test (n = 3 cultures/western blot group).

In cells without TBHP treatment, the PKCε activator DCPLA-ME did not affect PKCε, MnSOD, and VEGF mRNA expression (Figures 1D–F) but increased their protein translation (Figures 2B,D,F,J). In cells treated with TBHP, DCPLA-ME prevented the TBHP-induced decrease in MnSOD mRNA expression (Figure 1E). When compared with controls, bryostatin or DCPLA-ME in cells treated with TBHP did not increase PKCε, MnSOD, and VEGF mRNAs (Figures 1D–F) but increased their protein expression (Figures 2B,D,F,H,J,L). The results suggest that PKCε activation may promote PKCε, MnSOD, and VEGF protein expression without the increase in their mRNA expression.

### Effect of the Reactive Oxygen Species Scavengers on the Tert-Butyl Hydroperoxide-Induced Decrease in Manganese Superoxide Dismutase mRNA and Protein Expression

To verify whether the oxidative damage affect MnSOD mRNA and protein expression, cultured cells were incubated with the reactive oxygen species (ROS) scavenger *N*-acetylcysteine (Nac) or the cell-permeable SOD mimetic manganese (III) tetrakis(1-methyl-4-pyridyl)porphyrin (MnTMPyP) (Sen et al., 2018). Effect of the superoxide scavenger Nac and the superoxide dismutase mimetic drug MnTMPyP was studied in cultured cells treated with 500 μM TBHP for 1 h and maintained in culture medium for 3 days. Nac and MnTMPyP inhibited the effect of TBHP on the decrease in MnSOD protein expression, as determined with immunohistochemistry (Figures 3A,B) and western blot analysis (Figures 3C,D). Nac and MnTMPyP also blocked the TBHP-dependent decrease in MnSOD mRNA expression (Figure 3E). The results suggested that treatment with 500 μM TBHP for 1 h increases ROS production and oxidative stress that decreases MnSOD mRNA expression.

**FIGURE 3:** Reactive oxygen species (ROS) affects MnSOD mRNA and protein expression in cultured human brain microvascular endothelial cells (HBMEC) treated with tert-butyl hydroperoxide (TBHP). Cultured cells were incubated with the ROS scavenger *N*-acetylcysteine (Nac, 5 mM for 15 h) or the cell-permeable SOD mimetic manganese (III) tetrakis(1-methyl-4-pyridyl)porphyrin (MnTMPyP, 25 μM for 45 min) and were then treated with TBHP at 500 μM for 1 h and recovered without TBHP, Nac, and MnTMPyP for 3 days. **(A,B)** Immunohistochemistry and **(C,D)** western blot analysis were used to study MnSOD protein expression. **(E)** Quantitative PCR (qPCR) was used to determine MnSOD mRNA expression. Data are reported as mean ± SEM. Asterisks over the bars (*p < 0.05; **p < 0.01; ***p < 0.001) compared with their according controls, set as 100%. Student’s *t*-test for mRNA expression and western blot analysis (*n* = 4–5 cultures/group) or one-way ANOVA with *post hoc* Tukey’s multiple comparison test for immunohistochemistry (*n* = 42–160 random cells from 3 to 4 cultures per group).

### Effect of the PKCε-Dependent mRNA-Stabilizing Protein HuR on Manganese Superoxide Dismutase and Vascular Endothelial Growth Factor Expression

The HuR inhibitors dihydrotanshinone-I (DHTS) and CMLD-2 were used to study whether PKCε activated the mRNA stabilizing protein HuR, leading to the promotion of MnSOD and VEGF expression (Lal et al., 2017; Allegri et al., 2019). To investigate whether PKCε can activate HuR that can bind and chaperone the mRNA from the nucleus to the cytoplasm, immunohistochemistry was used to study the export of HuR from the nucleus to the cytoplasm during the PKCε activation (Figure 4A). Bryostatin and DCPLA-ME decreased the nuclear HuR per cytoplasmic HuR ratio compared to the control level, indicating that PKCε activation is associated with the nuclear export of HuR. The nuclear export of HuR was inhibited with the interfere of the specific binding of HuR to the ARE-binding sites in the mRNAs by the DHTS and CMLD-2 (Figure 4A).

**FIGURE 4:** The mRNA-stabilizing protein HuR involved in PKCε-activated MnSOD and VEGF expression in human brain microvascular endothelial cells (HBMEC). HBMEC cells were treated with the HuR inhibitor CMLD-2 (35 μM) or dihydrotanshinone-I (DHTS, 10 μM) for 30 min before and during the 3-day incubation in the presence of the PKCε activator bryostatin (25 nM) or DCPLA-ME (100 nM). **(A)** Immunohistochemistry of HuR was used to study nuclear export of the HuR protein. **(B)** Immunohistochemistry and **(C,D)** western blot analysis of MnSOD protein expression. **(E)** Quantitative PCR (qPCR) of MnSOD mRNA expression. **(F)** Immunohistochemistry and **(G,H)** western blot analysis of VEGF protein expression. M, molecular weight marker. Data are represented as mean ± SEM, *p < 0.05; ***p < 0.001; one-way ANOVA and *post hoc* Tukey’s multiple comparison test (*n* = 59–134 MnSOD-immunostained cells or 451–907 PKCε or VEGF-immunostained cells from 3 to 4 cultures/group or *t*-test (*n* = 3 cultures/western blot group).

Protein expression was studied with immunohistochemistry (Figures 4B,F) and western blotting, while change in mRNA expression was studied with qPCR (Figures 4C,D,G,H). The HuR inhibitors, DHTS and CMLD-2, significantly suppressed the PKCε-activated increase in MnSOD protein (Figures 4B–D) as well as mRNA expression (Figure 4E). DHTS and CMLD-2 also inhibited the PKCε-activated increase in VEGF expression (Figures 4F–H). The results indicate that posttranscription effect of PKCε on the increase in MnSOD and VEGF expression.

### Effect of the PKCε Activator in Rat Hippocampus With Age-Related Memory Impairment

Rats were trained with water maze swim learning for 5 days. For learning acquisition, aged (24 months old) rats with learning impairment exhibited increased swimming (latency) time to reach the hidden platform compared to young (5 months old) adult rats (Figure 5A). Age-related learning impairment was improved by bryostatin or DCPLA-ME treatment starting on day 3 of swim learning (Figure 5A). At 24 h after the final training swim, all animals underwent a probe test to evaluate whether they remembered the location of the platform despite being removed from the test area (Figure 5B). Age-related memory-impaired rats had poor memory to swim across to the removed platform site in the water maze compared to young rats (Figure 5B). Bryostatin and DCP-LA increased spatial memory to the young control level (Figure 5B).

**FIGURE 5:** The PKCε activator prevents spatial memory impairment and a decrease in vascular PKCε and MnSOD in the CA1 hippocampal stratum radiatum from aged rats. Age-related learning impairment rats (>24 months old) were injected with the PKCε activator bryostatin (bry, 5 μg/kg body weight) or DCP-LA (DCP, 1.5 mg/kg) diluted with normal saline, i.p., every other day for five injections before and three more injections during spatial memory training, compared to young (5 months old) and aged rats injected with normal saline (in the absence of the PKCε activator). Rats were trained with water maze to learn to find underwater platform for 5 days (2 swims/day). At 24 h thereafter, memory was determined how rats concentrated on the target area of the removed platform. **(A)** learning acquisition and **(B)** memory retention in aged rats, compared to control young rats. The learning and memory defect and MV loss were improved with the PKCε activator bryostatin and DCP-LA. **(C,E)** Colocalization of histochemistry of the vascular endothelium marker IB4 and immunohistochemistry was used to determine **(D)** PKCε and **(F)** MnSOD. Data are presented as mean ± SEM; *p < 0.05; **p < 0.01, ***p < 0.001; one-way ANOVA and *post hoc* Tukey’s multiple comparison test (*n* = 7–15 rats for behavioral study [2 swims/day/rat and 1 probe test/rat] or 63–95 random MV cells or 32–119 random areas from 3 to 5 rats/group).

We studied MV density in the hippocampal CA1 stratum radiatum using the isolectin B4 (IB4), which specifically binds terminal α-galactosyl residues of vascular endothelial cells to stain MV endothelium (Laitinen, 1987; Benton et al., 2008). Confocal microscopy was used to quantify immunostained levels of PKCε, MnSOD, and VEGF; each of them was colocalized with the vascular endothelial the isolectin B4 (IB4), which specifically binds terminal α-galactosyl residues of vascular endothelial cells (Laitinen, 1987; Benton et al., 2008), bound with biotin/avidin/green fluorescence dye complex (Figures 5C,E, 6A). PKCε, MnSOD, and VEGF were decreased in the MV endothelium in age-related memory-impaired rats compared to control young rats (Figures 5D,F, 6B). Bryostatin abolished the aging-dependent reduction in PKCε to the young control level (Figure 5D). For the effect related to oxidative stress, bryostatin treatment also rescued the aging-dependent decreases in MnSOD and even increased MnSOD higher than the level in young rats (Figure 5F). For the effect on angiogenesis, the reduction of VEGF in aged rats was reversed with bryostatin treatment (Figure 6B). We studied MV density using the IB4 at low magnification confocal microscopy. Change in MV density was determined with quantification of the IB4 area within hippocampal CA1 stratum radiatum (Figure 6C). Blood vessels decreased in age-associated memory-impaired rats (Figure 6D). The MV loss was rescued in the hippocampus by bryostatin and DCP-LA compared to aged rats without bryostatin or DCP-LA (Figure 6D). The results suggest that the decrease in PKCε, MnSOD, and VEGF expression in MV endothelium is associated with the MV loss during age-related memory impairment. The PKCε activators bryostatin and DCP-LA increase MnSOD and VEGF levels and MV density in aged rats with memory impairment.

**FIGURE 6:** The PKCε activator prevents a decrease in vascular VEGF and MV loss in the CA1 hippocampal stratum radiatum from age-related memory impairment rats. Tissue sections from rats in Figure 5 were used to stained with cytochemistry of the vascular endothelial cell marker IB4. **(A)** Colocalization of histochemistry of the vascular endothelium marker IB4 and **(B)** immunohistochemistry VEGF levels. **(C)** Low magnification of confocal microscope of the vascular endothelium marker IB4 was used to determine **(D)**. MV density in random hippocampal CA1 areas. Data are presented as mean ± SEM; **p < 0.01, ***p < 0.001; one-way ANOVA and *post hoc* Tukey’s multiple comparison test (*n* = 63–95 random MV cells or 32–119 random areas from 3 to 5 rats/group).

### PKCε, Manganese Superoxide Dismutase, and Vascular Endothelial Growth Factor mRNA and Protein Levels and Microvascular Density in Human Autopsy-Confirmed Alzheimer’s Disease Hippocampus

Autopsy-confirmed AD brains were collected between 6.83 and 28 h post-mortem (Table 1). No significant difference between post-mortem interval and immunohistochemistry (each primary antibody) was seen using linear regression analysis (not shown), suggesting that our results were not affected by post-mortem change within 28 h. The age was 79.4 ± 9.9 (mean ± S.E) years for AD brains, compared to 78.7 ± 11.4 years for age and gender-matched control (AC) brains. The Braak staging was 4.3 ± 0.4 (range = II–VI) for AD brains, compared to 1.4 ± 0.2 (range = 0–III) for AC brains.

**TABLE 1:** Demographic data of human brains.

Diagnosis	Braak	Age (year)	Gender	PMI (h)
Control Control Control Control Control Control Control Control Control Control Control AD AD AD AD AD AD AD AD AD AD AD AD AD	0 I I I I I I II II II III II II/III II/III III/IV IV IV V V V V V V VI	61 69 73 75 76 81 82 84 86 97 89 72 80 71 83 88 98 61 68 73 81 82 80 87	F M M F M F F F M M F M M M F F M F M F F F M M	16.80 18.43 20.88 20.08 12.25 26.18 15.70 19.25 25.28 17.00 14.12 6.83 23.17 28 5.9 16.67 22.70 21.42 15.67 17.67 20.75 18 15 15.25
				

Changes in PKCε, MnSOD, and VEGF were studied in AD subjects (*n* = 11) and AC controls (*n* = 11). AC control data were set at 100%, and all other experiment data were defined as% of their AC controls. qPCR was used to determine change in mRNAs at the whole hippocampal level. The PKCε and MnSOD mRNAs were reduced in the AD hippocampus compared to the AC control (Figures 7A,D). Immunohistochemistry and confocal microscopy were used to determined protein changes in the MV endothelium in the hippocampal CA1 stratum radiatum (Figures 7B,E). In parallel to changes in mRNA expression at the whole hippocampal level, MV endothelium in the hippocampus showed a decrease in PKCε and mitochondrial MnSOD levels (Figures 7C,F). The results indicate that AD pathogenesis is involved in the damage of PKCε and MnSOD mRNA expression, resulting in a decrease in PKCε and MnSOD translation.

**FIGURE 7:** Reduction of PKCε and mitochondrial MnSOD mRNA and protein expression in the CA1 stratum radiatum of autopsy-confirmed AD human hippocampus. **(A,D)** Quantitative PCR (qPCR) was used to detect PKCε mRNA at the whole hippocampus level and **(B,C,E,F)** immunohistochemistry and confocal microscopy were used to determine protein expression in MV wall cells in hippocampal CA1 area (N, the nucleus of MV wall cell). **(A)** mRNA and **(B,C)** protein expression for PKCε. **(D)** mRNA and **(E,F)** protein expression for MnSOD. AC, age-matched control; AD, autopsy-confirmed Alzheimer’s disease. PKCε and MnSOD mRNA and protein expression were reduced in overall AD brains (Braak stages II–VI), compared to AC controls (Braak stages 0–III). Data are reported as mean ± SEM, *p < 0.05; ^**^p < 0.01; ^***^p < 0.001; two-tailed *t*-test compared with their according controls (*n* = 11 hippocampi per group for qPCR or *n* = 182–365 random MV cells from 11 hippocampi per group).

Although VEGF mRNA was not changed in AD hippocampi (Figure 8A), VEGF protein expression in the MV wall cells was reduced in the AD hippocampi at Braak stages II-III, but not AD stages IV-VI, compared to the AC controls (Braak stages 0-III, Figures 8B,C). This suggests that AD pathogenesis is associated with decreased VEGF synthesis and/or increased VEGF degradation. Using immunohistochemistry of the vascular endothelial marker PECAM-1/CD31, overall MV area density was determined as % of MV fraction in random areas of the hippocampal CA1 radiatum (Figure 8D). The MV area in the AD hippocampi was decreased at Braak stages II-III, but not Braak stages IV-VI (Figure 8E). The results indicate that a decrease in PKCε, MnSOD and VEGF expression and the loss of microvessels is associated with AD pathogenesis.

**FIGURE 8:** Reduction of VEGF protein, but not mRNA, expression and microvascular loss in the CA1 stratum radiatum of autopsy-confirmed AD human hippocampus. **(A)** Quantitative PCR (qPCR) was used to detect VEGF mRNA at the whole hippocampus level. **(B,C)** Immunohistochemistry and confocal microscopy were used to determine VEGF protein expression in MV wall cells in hippocampal CA1 area (N, the nucleus of MV wall cell). **(D,E)** Immunofluorescence of the vascular endothelial cell marker CD31/PECAM was used to determine MV density. AC, age-matched control; AD, autopsy-confirmed Alzheimer’s disease. Although VEGF mRNA was not different among the experiment groups, VEGF and MV density was decreased in AD hippocampi at the early Braak stages II–III, but not AD at the late Braak stages IV–VI, compared to AC group. Data are reported as mean ± SEM, *p < 0.05; **p < 0.01; two-tailed *t*-test compared with their according controls (*n* = 11 hippocampi per group for qPCR or *n* = 182–365 random MV cells from 11 hippocampi per group, or 87–105 random CA1 areas from 5 AD Braak II–III, 14 AD Braak IV–VI and 19 AC).

### Effect of the PKCε Activator on Vascular Manganese Superoxide Dismutase and Vascular Endothelial Growth Factor in the Hippocampi of Alzheimer’s Disease Transgenic Mice Tg2576

Function effect of PKCε was studied in animal models treated with the PKCε activator drug, bryostatin. The effect of PKCε on MV density, VEGF, and MnSOD was studied in Tg2576 transgenic AD mice that overexpress a mutant form of APP (isoform 695) with the Swedish mutation (KM670/671NL). Double immunohistochemistry and confocal microscopy were used to evaluate PKCε, PKCα, MnSOD, and VEGF levels in vascular endothelial cells marked with platelet endothelial cell adhesion molecule (PECAM-1) or cluster of differentiation 31 (CD31) (Figures 9A,D, 10A).

**FIGURE 9:** The PKCε activator protects a reduction of PKCε and MnSOD in the hippocampal CA1 area from Tg2576 transgenic AD mice. Mice at 2 months of age were injected (i.p., twice a week) with normal saline in the presence or absence of bryostatin (30 μg/kg body weight) for a 3-month period. Mice were then studied at the age of 5–6 months old when an increase in soluble amyloid-beta (Aβ) and memory defect were seen in the hippocampus of Tg2576 mice (Hongpaisan et al., 2011). Bryostatin was withdrawn for 2 weeks to avoid the acute effect of bryostatin. Double immunohistochemistry and confocal microscopy of **(A,B)** PKCε, **(A,C)** PKCα, and **(D,E)** MnSOD in vascular endothelial cells that were marked with PECAM/CD31. Bryostatin (bry) prevented the loss of PKCε and MnSOD and promoted PKCα in Tg2576 (Tg) mice. Data are represented as mean ± SEM, *p < 0.05; ***p < 0.001; one-way ANOVA and *post hoc* Tukey’s multiple comparison test. (*n* = 35–74 random MV cells from 3 to 5 mice/group).

**FIGURE 10:** The PKCε activator protects a reduction of VEGF in MV endothelial cells and MV density in the hippocampal CA1 area from Tg2576 transgenic AD mice. Tissue sections from animals in Figure 9 were used. **(A)** Double immunohistochemistry and confocal microscopy of **(B)** VEGF in vascular endothelial cells that were marked with PECAM/CD31. **(C)** Cytochemistry of the vascular endothelial cells marker IB4, imaged with a confocal microscope, was used to determine **(D)** MV density in random CA1 areas. Bryostatin (bry) prevented the loss of VEGF and MV density in Tg2576 (Tg) mice. Data are represented as mean ± SEM, **p < 0.01; one-way ANOVA and *post hoc* Tukey’s multiple comparison test. (*n* = 35–74 random MV cells or 19–28 random areas from 3 to 5 mice/group).

Because bryostatin is a potent activator of PKCε and to a lesser extent PKCα (Hongpaisan and Alkon, 2007), changes in PKCε and PKCα were determined. Compared to the wild-type control mice, PKCε level in Tg2576 mice was decreased in MV endothelial cells that were treated with bryostatin (Figures 9A,B). Although PKCα concentration was not changed in Tg2576 mice, bryostatin significantly increased PKCα (Figures 9A,C). MnSOD was decreased in MV endothelial cells in Tg2576 mice compared to wild-type controls (Figures 9D,E). Treatment with bryostatin prevented the decrease in MnSOD (Figures 9D,E).

We further determined change of VEGF level. Compared to wild-type littermate sibling mice, a reduction of VEGF in MV endothelial cells in Tg2576 mice was prevented after bryostatin treatment (Figures 10A,B). IB4 histochemistry was used to determine MV density (Figure 10C). The PKCε activator bryostatin prevented the MV loss in Tg2576 mice (Figure 10D). Taken together, the results suggest that the PKCε activator can prevent the decrease in PKCε MnSOD and VEGF levels and in MV loss in AD transgenic mice Tg2576.

## Discussion

The present study demonstrated that the TBHP-induced short-term oxidative stress decreased MnSOD—but not PKCε and VEGF—mRNA and protein expression in cultured HBMEC cells that were blocked by superoxide degrading drugs, Nac and MnTMPyP. The PKCε can increase PKCε mRNA and its protein expression and increase MnSOD mRNA, MnSOD, and VEGF expression, promoted by the mRNA-stabilizing protein HuR that bind ARE sequence in MnSOD and VEGF mRNAs. Under chronic conditions in animal models, reduced PKCε was associated with a decrease in MnSOD and VEGF expression in MV endothelial cells and MV density in the hippocampi of aged rats (>24 months old) and young AD transgenic mice Tg2576 (5–6 months old). The PKCε activators DCP-LA and bryostatin rescued the reduction of PKCε, MnSOD, and VEGF in MV cells and the MV loss.

During the aging process, the activity of sirtuin1 (SIRT1) in the nucleus is reduced, which decreases the von Hippel-Lindau (pVHL) protein levels and subsequently stabilizes hypoxia-inducible factor-1α (HIF-1α). Activated HIF-1α reduces the proliferator-activated receptor-gamma coactivator 1β (PGC-1β) activity, resulting in the downregulation of mitochondrial genes and MnSOD (Lu et al., 2010; Yeo, 2019). c-Myc activity is also inhibited upon its interaction with HIF-1α. c-Myc targets gene-regulating processes required for cell growth, including rRNA transcription and processing, ribosomal protein transcription and translation, and translation initiation (Lu et al., 2010). The reduction of c-Myc activity may elicit the loss of VEGF (Baudino et al., 2002; Florea et al., 2013). In the present study, it is likely that the PKCε activator may have increased SIRT1 and c-Myc, resulting in the increase in MnSOD mRNA transcription during oxidative stress (Li et al., 1996; Thompson et al., 2013).

In the present study, normal aging and AD pathogenesis were associated with a decrease in PKCε, MnSOD, and VEGF, possibly due to a prolonged and significant increase in O_2_^•–^ that favors reaction with the free radical nitric oxide (NO^⋅^) to form peroxynitrite (ONO_2_^–^), a powerful oxidant that damages DNA, RNA, and proteins, including PKC (Maher, 2001). On the other hand, the PKCε activator can restore the mitochondria antioxidant MnSOD that may buffer oxidative stress and may inhibit the oxidative damage of PKCε and VEGF. It has been previously shown that the PKCε activators can increase PKCε itself; however, the mechanism is not clearly understood (Hongpaisan et al., 2011, 2013).

In a previous study, we showed that DCP-LA and/or bryostatin improved recent memory retention, which is important for daily living activity, by restoring the reduction of PKCε accumulation in axonal and presynaptic axonal boutons and improving synaptic formation/modification in aged rats and AD transgenic mice Tg2576 and 5xFAD. This was done by preventing/improving PKCε-activated mRNA-stabilizing protein HuD or ELAV-like protein 4, which inhibits mRNA degradation and promotes MnSOD and BDNF in hippocampal neurons (Hongpaisan et al., 2011, 2013; Sen et al., 2018). PKCε is critical in synaptogenesis and memory (Prekeris et al., 1998; Aranda-Abreu et al., 1999; Hama et al., 2004), and the present study demonstrated that DCPLA and bryostatin can rescue the loss of blood vessels by preventing and/or restoring the loss of PKCε, MnSOD, and VEGF that may contribute to improved learning acquisition and memory retention in animal models of normal aging (as shown in the present study) and AD transgenic mice Tg2576 and 5xFAD (Hongpaisan et al., 2011, 2013; for review see Govoni et al. (2010), Talman et al. (2016)).

In the present study, the mRNA-stabilizing protein HuR is involved in the effect of PKCε activator by suppressing MnSOD and VEGF mRNA degradation. PKCε may stimulate protein phosphatase 2A (PP2A) to facilitate the dephosphorylation of phospho-Akt and subsequently lead to the accumulation of the dephosphorylated and active forkhead box O3s (FOXO3a), which activates MnSOD mRNA transcription, while PKCα may phosphorylate the CREB transcription of MnSOD mRNAs (Chung et al., 2011). Binding of VEGF on vascular endothelial growth factor receptor 2 (VEGFR2) can activate the PKC/extracellular signal-regulated kinase (ERK) 1/2 signal cascade. In the present study, the PKCε activator may therefore promote VEGF signaling by directly activating extracellular signal-regulated kinase (ERK) 1/2 and vascular proliferation (Rask-Madsen and King, 2008).

## Conclusion

During aging and AD pathogenesis, PKCε, MnSOD, and VEGF expression decreases in MV endothelial cells and MV loss occurs in the hippocampus. The PKCε activators can reduce the decrease of PKCε and MnSOD mRNA and protein expression in MV cells. PKCε activators can also increase VEGF, which is important for angiogenesis and blood vessel maintenance.

## Data Availability Statement

The original contributions presented in the study are included in the article, further inquiries can be directed to the corresponding author.

## Ethics Statement

The animal study was reviewed and approved by Institutional Animal Care and Use Committee at Thomas Jefferson University.

## Author Contributions

JH: conceptualization and writing – original draft. GM, HW, ZZ, and JH: formal analysis. GM, HW, ZZ, DA, and JH: writing – review and editing. All authors contributed to the article and approved the submitted version.

## Conflict of Interest

DA was employed by Neurotrope Bioscience, Inc. The remaining authors declare that the research was conducted in the absence of any commercial or financial relationships that could be construed as a potential conflict of interest.

## Publisher’s Note

All claims expressed in this article are solely those of the authors and do not necessarily represent those of their affiliated organizations, or those of the publisher, the editors and the reviewers. Any product that may be evaluated in this article, or claim that may be made by its manufacturer, is not guaranteed or endorsed by the publisher.

## Footnotes

1
http://www.wma.net/en/30publications/10policies/b3/index.html

2
http://rsb.info.nih.gov/ij/
